# Study on the Mechanism of Cardiac Intensive Care after Thoracoscopic Surgery

This article has been retracted.

**DOI:** 10.1155/2022/2894755

**Published:** 2022-03-30

**Authors:** Min Lin, Maoting Ye, Jing Ren

**Affiliations:** The First Affiliated Hospital of Army Medical University, Chongqing 400000, China

## Abstract

**Objective:**

To explore the mechanism of intensive care of the heart after thoracoscopic surgery.

**Methods:**

104 patients with severe cardiac disease were selected after thoracoscopic surgery in our hospital, received nursing care after surgery, and divided into control group (*n* = 53) and research group (*n* = 51) according to different nursing methods. Before nursing, the research group carried out targeted nursing and prevention of postoperative complications. The quality of life, complications, anxiety, depression and satisfaction scores, 6-minute walking distance, self-care ability scores, and cardiac function were compared between the two groups.

**Results:**

Patients' quality of life scores improved significantly in both groups after treatment, but the increase was greater in the study group than in the control group (*P* < 0.05); the incidence of complications was 18.9% and 5.9% in the study and control groups, respectively, and the incidence of complications was lower in the study group than in the control group (*P* < 0.05); and the incidence of complications was lower in the study group than in the control group (*P* < 0.05). After care, patients' anxiety and depression scores were significantly lower, and satisfaction scores were significantly higher in both groups, with a greater change in the study group than in the control group (*P* < 0.05); after care, patients' 6-minute walking distance was significantly higher in both groups, with a greater change in the study group than in the control group (*P* < 0.05); after care, LVEF indicators were significantly higher, and LVESD and LVED indicators were significantly higher, with a greater change in the study group than in the control group. After care, LVEF indexes increased significantly in both groups, while LVESD and LVED indexes decreased significantly in the study group, with a greater change than in the control group (*P* < 0.05); after care, systolic blood pressure and heart rate increased significantly in both groups, with a greater increase in the study group than in the control group (*P* < 0.05); after care, systolic blood pressure and heart rate increased significantly in both groups, with a more significant increase.

**Conclusion:**

Targeted nursing for patients with severe cardiac disease after thoracoscopic surgery has a significant effect, which can improve patients' anxiety and depression, significantly improve patients' self-care ability and quality of life, and at the same time improve patients' cardiac function, heart rate, and blood pressure, with high patient satisfaction.

## 1. Introduction

Thoracoscopic surgery is widely used in clinical practice and is a new technology for the treatment of cardiovascular disease. Thoracoscopic surgery can change the traditional development mode of cardiac surgery and currently plays an important role in the surgical treatment of various cardiac diseases [1]. Nonetheless, thoracoscopic cardiac surgery can also trigger a stress response, which threatens the patient's normal life to a large extent. Therefore, the current postoperative prognosis of patients should be highly valued, and timely intervention measures should be taken to reduce the incidence of complications [2].

In this study, 104 patients with severe cardiac disease after thoracoscopic surgery in our hospital were selected, targeted nursing care was given to the patients, and postoperative complications were prevented, and the nursing mechanism of 104 patients with severe cardiac disease after thoracoscopic surgery was explored. The contents are as follows.

## 2. Materials and Methods

### 2.1. General Information

The patients were divided into two groups: control group (*n* = 53), 28 males and 25 females, aged 30-82 years, average age of 53.8 ± 4.2, duration of disease 1-8 years, and average of 3.7 ± 1.2 years, including 32 cases of coronary heart disease and 21 cases of myocardial infarction, and study group (*n* = 51), 27 males and 24 females, aged 30-81 years, average age of 53.6 ± 4.1), and duration of disease 1-8 years. In the study group (*n* = 51), there were 27 males and 24 females, aged 30-81 years, mean age of 53.6 ± 4.1, duration of disease 1-8 years, and mean of 3.5 ± 1.3 years, including 30 cases of coronary artery disease and 21 cases of myocardial infarction. The study subjects agreed to the study; the data were comparable (*P* > 0.05) and approved by the hospital ethics committee.

Inclusion criteria are as follows: ① patients with high compliance and normal cognitive function; ② patients with stable vital signs and acceptable for prognostic follow-up; and ④ patients who meet the criteria for severe cardiac disease after thoracoscopic surgery and who met the criteria for laparoscopic cardiac stenting intervention. Exclusion criteria are as follows: ① patients with contraindications to surgery; ② patients with abnormal coagulation or liver and kidney function; ③ patients with other organ diseases; and ④ patients during pregnancy or breastfeeding.

### 2.2. Methods

Patients' vital signs, such as respiration, body temperature, heart rate, and blood pressure, were monitored in the control group, as were skin mucous membrane color and mental changes, postoperative fluid intake and output were recorded, the volume, nature, and color of urine were observed in the early postoperative period, and if abnormalities occurred, the doctor was immediately notified for active treatment and intervention.

The study group got tailored treatment and postoperative complication prevention.

1. Psychological care: medical workers actively interacted with patients to better understand their emotional changes. Patients are questioned about postoperative pain following the surgery and warnings are provided. If the patient is suffering anxiety or depression, the healthcare staff should console him or her as quickly as possible, eliminate any fear or concern, and encourage the patient to boost his or her motivation for treatment
2. Nutritional care: provide dietary recommendations to patients and design a meal plan. Give a high-vitamin, high-calorie, and high-protein diet, utilize more readily digested meals, decrease salt and fat consumption, and ban stimulating foods
3. Insomnia prevention: patients' postoperative unfavorable emotions likely have an influence on sleep quality and should be supplemented with psychological treatment to offer timely consolation to patients and keep them happy. If the patient's blood pressure is normal and there is no postoperative bleeding at the puncture site, the bodyweight should be changed to the healthy side and the calf on the operated side should be relaxed suitably to reduce the pain. To establish a suitable resting environment for the patient, prohibit visits at night and decrease the sound of corridor strolling and instruments
4. Preventing hemorrhage and local hematomas: too little compression at the puncture site or the use of intraoperative anticoagulants might result in bleeding and edema at the puncture site; consequently, healthcare workers should apply sandbag compression at the puncture site to avoid wound bleeding. In addition, the puncture site should be evaluated 48 hours following surgery, and the patient should be able to get out of bed if there are no hard knots, seeping, or bleeding. Otherwise, patients should not be permitted to get out of bed too early and should notify their doctor right away if they have any strange symptoms
5. Prevention of hypotension and vagal reflexes: inadequate preoperative rest, nervousness, and prolonged fasting are the main causes of abnormal vagal reflexes. Medical staff should provide positive psychological care to relieve the patient's tension. They should also shorten the preoperative fasting period, ensure that the patient has sufficient sleep and rest, and monitor the patient's electrocardiogram, heart rate, and blood pressure. In addition, preoperative therapeutic devices and medications should be prepared, and the number of fluid drops should be adjusted according to the patient's cardiac function status
6. Urinary retention prevention: urinary retention issues can be caused by prolonged surgical bed rest, wound discomfort, or unfamiliar peeing in bed. Before surgery, the patient should be taught to defecate in bed so that he or she can become accustomed to it. Additionally, the patient should be urged to drink enough water or listen to the sound of flowing water to aid defecation and give as much privacy as possible to alleviate discomfort and strain. If the previous treatments fail, catheterization can be used to help with defecation; however, the volume of catheterization should be limited to 500 ml each time
7. Thromboprophylaxis: because of the length of the procedure and the impact of contrast and anesthesia on limb movement and consciousness, the patient's dorsalis pedis artery pulse should be monitored and anticoagulant medication should be administered. In addition, the patient should be given limb braking and massage to speed up blood circulation

### 2.3. Observation Indicators

#### 2.3.1. Quality of Life [3]

To assess a patient's physical, social, cognitive, and role functioning, use the SF-36 scale. Each function has a total score of 100 points. The greater the quality of life, the higher the score.

#### 2.3.2. Complications

Count the number of cases of insomnia, local hemorrhage or edema, urinary retention, vagus nerve reflex, and hypotension, and calculate the incidence.

- Depression, anxiety, and satisfaction scores [4]: assess patients' sadness and anxiety before and after therapy using the Hamilton Sadness Scale (HAMD) and Hamilton Anxiety Scale (HAMA). There are a total of 24 items, and the lower the score, the more depressed and anxious the person is. The lighter the material, the better. The patient's happiness was measured using our hospital's developed satisfaction test, which had a total score of 10 points. The higher the score, the happier the nurses
- 6-minute walking distance [5]: ask the patient to walk as hard as possible for 6 minutes, record the longest walking distance, and evaluate the patient's exercise ability and body endurance

#### 2.3.3. Self-Care Ability Score [6]

Contains four items: self-concept, self-care responsibility, self-care skills, and health knowledge level. The total score is 100 points. The higher the score, the stronger the patient's self-care ability.

#### 2.3.4. Cardiac Function [7]

Use cardiac color Doppler ultrasound to measure left ventricular ejection fraction (LVEF), left ventricular end-diastolic diameter (LVEDD), and left ventricular end-systolic pressure (LVES), according to the instructions.

### 2.4. Statistical Methods

The count data were described using the composition ratio and rate, the chi-square test was chosen for the analysis of variance between groups, the measurement data were expressed as mean standard deviation, the *t*-test was chosen for the analysis of variance between groups, and the body mass of the case groups was calculated if the data passed the normal distribution test.

Logistic regression analysis was used to investigate the important components, and a difference of *P* 0.05 was judged statistically significant. GraphPad Prism8 was the graphical application used in this investigation.

## 3. Results

### 3.1. The Two Groups' Quality of Life Scores Were Compared

Prior to treatment, there was no significant difference in physical, social, cognitive, or role functions between the two groups (*P* > 0.05). After treatment, both groups' quality of life scores improved considerably, with the study group improving more than the control group, and the difference between the two groups was statistically significant (*P* < 0.05) (Table 1).

### 3.2. Comparison of Complication Rates between the Two Groups

Complications occurred in 18.9% of the study group and 5.9% of the control group, respectively. The study group had a lower incidence of complications than the control group, and the difference was statistically significant (*P* < 0.05) when the two groups were compared (Table 2).

Prior to nursing, there was no significant difference between the two groups in terms of anxiety, depression, or satisfaction (*P* > 0.05). After nursing, both groups' anxiety and despair levels were much lower, and their satisfaction ratings were significantly greater. The modifications in the research group were more pronounced than in the control group. The difference between the two groups was statistically significant (*P* 0.05) (see Figure 1).

Before nursing, there was no significant difference in 6-minute walking distance between the two groups (*P* > 0.05). After breastfeeding, both groups' 6-minute walking distances rose considerably, with the study group changing more than the control group. There was a statistical difference between the two groups (academic significance: *P* < 0.05) (Figure 2).

The self-care skill evaluations of the two groups were compared. Before nursing, there was no significant difference in self-concept, self-care responsibility, self-care ability, or health knowledge level between the two groups (*P* > 0.05). After nursing, both groups' self-care skills increased significantly. The study group rose faster than the control group, with a statistically significant difference (*P* 0.05) between the two groups (Figure 3).

The LVESD, LVEF, LVED, and other cardiac function indicators were not significantly different between the two groups before breastfeeding (*P* > 0.05). The LVEF indices of both groups increased dramatically after nursing, but the LVESD and LVED indexes fell significantly according to the research team. The range of change was higher in the experimental group than in the control group, and the difference between the two groups was statistically significant (*P* < 0.05) (Figure 4).

Before nursing, there was no significant difference between the two groups in systolic blood pressure or heart rate (*P* > 0.05). Both groups' systolic blood pressure and heart rate rose considerably after nursing, with the study group's rise being greater than the control group. The difference was statistically significant (*P* 0.05) when compared to each other (Figure 5).

## 4. Discussion

Compared with traditional surgical treatment, patients are more accepting of thoracoscopic surgery [8]. Any operation, however, may be stressful and cause a range of problems, which can diminish the treatment's success rate, jeopardise the patient's prognosis, and, in extreme situations, even endanger the patient's life [9]. As a result, preventing problems and providing postoperative care are critical [10].

This study reduced the incidence of bleeding and local hematoma complications by sandbag compression of the puncture site [11]. The incidence of hypotension, vagal reflexes, and insomnia complications can be reduced by psychological care, shortening the duration of preoperative fasting and ensuring adequate sleep [12]. Complications of urinary retention can be prevented by training patients to defecate in bed, drinking more water, and listening to the sound of running water for bowel movements [13]. Thrombotic complications can be prevented by giving anticoagulants and limb massage [14]. The study's findings revealed that the study and control groups had complication rates of 18.9% and 5.9%, respectively, with the study group having a lower complication rate than the control group, and the difference between the two groups was statistically significant (*P* < 0.05). The findings of this study were consistent with those of Feng et al. [15]. The findings show that focused treatment may minimize the risk of complications more effectively than standard care and that psychological counseling and complication prevention can enhance surgical success rates and speed recovery. Patients' lack of awareness of illness causation and treatment concepts may lead to anxiety and sadness, which can disrupt surgery and have a negative impact on their recovery [16–18]. By actively communicating with patients in this study, healthcare professionals can understand the changes in patients' emotions and postoperative pain levels [18, 19] and can develop targeted care measures based on patients' specific conditions, which can play an important role in alleviating patients' negative emotions [19–21]. This research looked at how patients' moods changed before and after treatment. The study's findings revealed that there was no statistically significant difference in anxiety, depression, or satisfaction scores between the two groups before treatment (*P* > 0.05), but after treatment, anxiety and depression scores in both groups decreased significantly, while satisfaction scores increased significantly, with a greater change in the study group than in the control group, and the difference between the two groups was statistically significant (*P* < 0.05). The findings revealed that psychological care may enhance patients' self-confidence and treatment compliance, which can help patients overcome their concerns, improve their negative emotions, and boost their satisfaction with their care.

Self-care ability refers to the ability to care for oneself and conscious self-care activities. Self-care ability has an impact on patients' well-being and life health, and the nursing staff in this study were able to improve patients' self-care compliance and cooperation in complication prevention by talking about the surgery and precautions, which contributed to the overall outcome of the surgery. Patients' self-care capacity and quality of life ratings increased considerably in both groups after treatment, with the study group exhibiting a bigger rise than the control group, and the difference between the two groups was statistically significant (*P* < 0.05). The present results suggest that concentrated nursing interventions may improve patients' self-care skills after laparoscopic cardiac stenting operations and that patients' various daily functions and quality of life significantly improved. By monitoring vital indicators such as breathing, body temperature, heart rate, and blood pressure, as well as examining skin mucous membrane color and mental changes, the research was able to better protect patients' lives, allowing early action to be done in emergency scenarios. The study's findings revealed that following care, both groups' systolic blood pressure and heart rate were considerably higher, with the study group's rise being more apparent than the control group, and the difference was statistically significant when comparing the two groups (*P* < 0.05). The findings show that tailored nurse interventions can enhance patients' vital signs and speed up their recovery after surgery. This study explored the nursing mechanism and cardiac function changes of patients after thoracoscopic surgery. The study's findings revealed that following care, both groups' 6-minute walking distance rose considerably, with the study group's rise being bigger than the control group's ((P <0.05). The results show that dietary intervention for patients after thoracoscopic surgery can improve the patient's body tolerance and is beneficial to the improvement of cardiac function.

In conclusion, targeted nursing for patients with severe cardiac disease after thoracoscopic surgery has a significant effect, which can improve patients' anxiety and depression, significantly improve patients' self-care ability and quality of life, and at the same time improve patients' cardiac function, heart rate, and blood pressure, with high patient satisfaction.

## Figures and Tables

**Figure 1:** Comparison of anxiety, depression, and satisfaction scores between the two groups.

**Figure 2:** Comparison of the 6-minute walking distance between the two groups.

**Figure 3:** The self-care ability scores of the two groups were compared.

**Figure 4:** The two groups' cardiac functions were compared.

**Figure 5:** The systolic blood pressure and heart rate of the two groups were compared.

**Table 1:** Comparison of the two groups' quality of life scores (*x* ± *s*).

Group	Time	Somatic functions	Social functions	Cognitive functions	Character functions
Control group	Prenursing	63.2 ± 3.9	68.2 ± 3.8	62.8 ± 3.5	68.2 ± 3.3
	Aftercare	79.2 ± 4.4	76.9 ± 6.2	82.5 ± 4.1	82.6 ± 4.1
Research group	Prenursing	63.6 ± 4.1	68.1 ± 4.0	62.6 ± 3.4	68.4 ± 3.2
	Aftercare	90.5 ± 4.6	88.4 ± 5.3	92.4 ± 4.3	91.6 ± 4.5

Note: Within-group comparison, ^a^*P* < 0.05; between-group comparison, ^b^*P* < 0.05.

**Table 2:** Comparison of complication rates between the two groups (*x* ± *s*).

Group	Number of examples	Insomnia	Localised bleeding or edema	Urinary retention	Vagal reflex	Low blood pressure	Incidence
Control group	53	3 (5.7)	2 (3.8)	1 (1.9)	1 (1.9)	3 (5.7)	18.9%
Research group	51	2 (3.8)	1 (1.9)	0 (0.0)	0 (0.0)	0 (0.0)	5.9%
*X* ^2^	/	/	/	/	/	/	6.248
*P*	/	/	/	/	/	/	<0.05

## Data Availability

The data used to support the findings of this study are included within the article.
